RETRACTED

# Identification and Verification of Key Tumor Genes Associated with Diagnosis and Prognosis of Breast Cancer Based on Bioinformatics Analysis

**DOI:** 10.1155/2022/9041466

**Published:** 2022-05-31

**Authors:** Feng Yu, Xian-jun Pan, Jie Luo

**Affiliations:** Chongqing Key Laboratory of Translational, Research for Cancer Metastasis and Individualized Treatment, Chongqing University Cancer Hospital, Chongqing 400030, China

## Abstract

Breast cancer (BC) is the most common cancer and the most frequent cause of cancer death among women worldwide. The aim of the present study was to identify the critical genes for the diagnosis and prognosis of BC. Two mRNA expression data (GSE29431 and GSE42568) were acquired from the GEO database. The determination of differently expressed genes (DEGs) between BC specimens and nontumor specimens was completed via the LIMMA package of R. GO annotation and KEGG pathway enrichment analyses were applied to explore the function of DEGs. Kaplan-Meier methods were used to determine the prognostic value of DEGs in BC using TCGA datasets. The diagnostic value of the survival-related DGEs were confirmed using ROC assays in two GEO datasets. RT-PCR was used to examine the expression of the critical genes in BC cells and normal breast cells. CCK-8 experiments were applied to explore the function of the critical genes in BC cells. In this study, we identified 31 DEGs between BC specimens and nontumor specimens. KEGG analysis revealed 31 DEGs were involved in PPAR signal path, AMPK signal path, glycerolipid metabolism, adipocytokine signaling pathway, phenylalanine metabolism, tyrosine metabolic process, and glycine, serine, and threonine metabolic process. Four DEGs including CRYAB, DEFB132, MAOA, and RBP4 were observed to be associated with clinical outcome of BC patients. Their diagnostic values were also confirmed in both GSE29431 and GSE42568 datasets. In addition, we analyzed TCGA datasets and confirmed that the results were consistent with GEO datasets. Finally, the results of RT-PCR confirmed that the expression of CRYAB and RBP4 was distinctly downregulated in BC cells. CCK-8 analysis revealed that overexpression of CRYAB and RBP4 distinctly suppressed the proliferation of BC cells. Overall, our findings suggested CRYAB and RBP4 as critical genes for the diagnosis and prognosis of BC patients. They may be used as novel biomarkers for BC patients.

## 1. Introduction

Breast cancer (BC) is a leading cause of tumor-associated mortality in females across the globe [1]. Over the past 10 years, BC is characterized as a high prevalence and death rate in PRC [2]. From the perspective of histology, BC can be separately into four main subtypes, like HER2-enriched, luminal A, luminal B, and triple-negative [3]. Despite the fact that the amelioration in timely identification and therapy has reduced BC death rates recently, preventing and treating BC are still challenging [4, 5]. Hence, discovering more biomarkers to forecast the response of therapy, cancer development, and potential target therapies is becoming more and more important.

RETRACTED

Recent developments in microarray profiling and genome-wide sequencing have accelerated the identification of novel prognostic biomarkers that are important for precise classification of tumors and personalized treatment decisions [6, 7]. Substantial researches on early-stage BC have revealed that genome data produced from sufferers with long-term follow-up are better than the staging method nowadays in speculating prognostic results [8, 9]. In these researches, massive genes have been produced to categorize BC sufferers with diverse clinic results. Identification of novel diagnostic and prognostic biomarkers based on multiple datasets is very important [10, 11]. In this study, we analyzed GSE29431 and GSE42568 datasets to identify differently expressed genes (DEGs) in BC. Then, we further screen the survival-related DEGs using TCGA datasets. Finally, RT-PCR was completed to demonstrate the expressing of the survival-related DEGs in BC cell lines and finished CCK-8 analysis to investigate related functions.

## 2. Materials and Methods

### 2.1. Cell Lines and Cell Culture

One normal breast epithelium lineage cell (HBL-100) and 4 mankind BC lineage cells (BT-549, MDA-MB-468, MDAMB-231, and MCF-7) were provided by the Institution of Biological Chemistry and Cell Biology of Chinese Academy of Sciences (PRC). Cells were cultivated with DMEM (iCell-0003, iCell Biological Science, PRC) added with 100 U/mL penicillin/kyowamycin (Invitrogen, PRC) and 10% FBS (Gibco, PRC) in a humid cultivation chamber with 5% CO_2_ under 37°C.

### 2.2. Cell Transfection

A full-length CRYAB and RBP4 sequence was synthesised and introduced into pcDNA3.1 vector via insertion (Invitrogen) to produce pcDNA3.1-CRYAB and pcDNA3.1-RBP4. Plasmid vectors (pcDNA3.1-CRYAB, pcDNA3.1-RBP4, and pcDNA3.1-NC) were produced via DNA Midiprep tools (Qiagen, Germany). When reaching approximately 80% confluence, MDA-MB-468 and BT-549 cells were subjected to plasmid vector transfection via liposome transfection reagent 2000 (Invitrogen) as per the recommendations of the supplier. Posterior to the 48 h transfectional process, cells were collected for subsequent assays.

### 2.3. Cell Proliferation Assay

Cellular proliferative ability was speculated via CCK-8 analysis (Dojindo, Japan). Overexpression transfected MDA-MB-468 and BT-549 were inoculated onto the 96-well dishes, and each was cultivated for 0 h, 24 h, 48 h, 72 h, and 96 h separately. At diverse temporal points, 10 *μ*L CCK-8 was supplemented into the well and cultivated for 120 min. An optical density (OD) of 450 nm was identified via a microplate reading device.

RETRACTED

### 2.4. Microarray Data

Two independent BC gene expression profiles (GSE29431 and GSE42568) were acquired from the GEO database (https://www.ncbi.nlm.nih.gov/geo/) and utilized as discovery datasets to determine DEGs. GSE29431 included 12 normal BC specimens and 54 BC specimens. GSE42568 included 17 normal BC specimens and 104 BC specimens. Every dataset was acquired from the microarray platform of Affymetrix Human Genome U133 Plus 2.0 Array [HG-U133_Plus_2]. Expression comparisons of 1101 breast tumors and 459 normal samples from TCGA and the GTEx projects were done using ACLBI (http://www.aclbi.com) tools.

### 2.5. DEG Determination

The determination of DEGs was completed via the LIMMA package of R. The adjusted *P* values (adj *P* value) were utilized to prevent the false-positive outcomes. Genes with |log2 fold change (FC)| and adj *P* < 0.01 were considered DEGs between cancers and nontumor samples. Ggplot2 and Venn Diagram packages of R were utilized to produce volcanic plot and Venn diagram, separately, for the visualisation of the determined DEGs.

### 2.6. Gene Ontology (GO) Annotation and the Kyoto Encyclopedia of Genes and Genomes (KEGG) Pathway Enrichment Analyses

For the sake of revealing the roles of DEGs, Enrichr database was utilized to complete GO analysis and KEGG analysis [12]. The GO terms comprised 3 aspects: biological process (BP), cellular component (CC), and molecular function (MF). Adj.*P* < 0.05 was regarded as statistically significant.

### 2.7. Diagnosis Significance of Feature Markers in BC

For the sake of testing the prediction significance of the determined markers, our team produced a ROC curve via the mRNA expression data from GSE29431 and GSE42568. The AUC value was employed to identify the diagnosis validity in the discrimination of BC specimens.

### 2.8. Statistical Analysis

Statistic assay was completed via R program (v 4.0.2) packages and SPSS 20.0 (SPSS, Chicago, IL, USA). Perl language was utilized for data matrix and the entire processing of data. The Student's *t*-test was utilized to study statistically significant diversities between groups. Differences were considered statistically significant when *P* < 0.05.

## 3. Results

### 3.1. Determination of DEGs in BC

To identify the potential biomarkers for BC, we analyzed GSE29431 datasets and identified 34 downregulated genes in BC specimens (Figure 1(a)). In addition, via analyzing GSE42568 datasets, we identified 60 downregulated genes and 10 upregulated genes in BC specimens (Figure 1(b)). Moreover, 31 overlapping genes were identified between GSE29431 and GSE42568 datasets (Figure 1(c) and Table S1). The above 31 genes may be involved in the progression of BC.

RETRACTED

### 3.2. Functional Enrichment Analysis of 31 DEGs

To explore the biofunction of 31 DEGs in BC, we perform GO and KEGG analyses using the ClusterProfile R package. The results showed that 31 DEGs were mainly involved in fatty acid metabolic process, modulation of lipometabolism, reaction to peptide hormone, reaction to monosaccharide, lipidic droplet, mitochondrial outer membrane, chylomicron, sperm head, carboxylic acid binding, monocarboxylic acid binding, growth factor binding, and hormone acceptor binding (Figure 2(a)). Meanwhile, KEGG analyses revealed that pathways were significantly sponged including PPAR signal path, AMPK signal path, glycerolipid metabolism, adipocytokine signaling pathway, phenylalanine metabolism, tyrosine metabolic process, and glycine, serine, and threonine metabolic process (Figure 2(b)). Our findings suggested that the 31 DEGs may be involved in the progression of tumors.

### 3.3. Identification of Survival-Related DGEs in BC Using TCGA Datasets

To identify survival-related DGEs in BC, we analyzed TCGA datasets based on 31 DEGs in GSE29431 and GSE42568 datasets. As shown in Figure 3(a), only 4 genes including CRYAB, DEFB132, MAOA, and RBP4 were identified to be survival-related DGEs in BC patients. Moreover, we also confirmed that the expression of CRYAB, DEFB132, MAOA, and RBP4 was distinctly downregulated in BC patients compared with nontumor specimens from TCGA datasets (Figure 3(b)). Moreover, we performed ROC assays based on GSE29431 and GSE42568 datasets. Importantly, we observed that all four genes showed a strong ability in screening BC specimens from nontumor specimens (Figures 4(a) and 4(b)).

### 3.4. The Oncogenic Roles of RBP4 in BC

To further demonstrate the expression of CRYAB, DEFB132, MAOA, and RBP4 in BC, we performed RT-PCR using four BC cells and HBL-100. As shown in Figure 5(a), the expression of DEFB132 and MAOA remained unchanged between BC specimens and healthy samples. However, our team observed that the expression of CRYAB and RBP4 was distinctly downregulated in BC specimens and nontumor specimens (Figure 5(b)). Next, we observed that MDA-MB-468 and BT-549 cells transfected with pcDNA3.1-CRYAB and pcDNA3.1-RBP4 exhibited significantly increased CRYAB and RBP4 expression (Figure 5(c)). Moreover, we performed CCK-8 assays to explore the possible functions of overexpression of CRYAB and RBP4 on cellular proliferation. As shown in Figure 5(d), overexpression of CRYAB did not influence the proliferative capability of MDA-MB-468 and BT-549 cells. However, overexpression of RBP4 was observed to suppress the proliferative ability of MDA-MB-468 and BT-549 cells (Figure 5(e)). Thus, RBP4 might be a new treatment target for BC.

RETRACTED

## 4. Discussion

BC is the most common malignant tumor in females across the world [13, 14], despite the fact that the quantity of BC survivors is increasing because of timely diagnoses and ameliorated therapeutic regimens [15, 16]. Nevertheless, the quantity of females experiencing relapse related to unexpected prognoses posterior to the diagnoses of the primary cancer, like metastasis and unsatisfactory life quality, is elevating as well [17, 18]. Hence, the determination of noninvasive biological markers with remarkable sensitiveness and specificness for timely BC identification and the surveillance of the responsiveness to treatment is essential for the amelioration of prognoses. In the present research, our team intended to determine new biological markers for BC based on GEO and TCGA datasets.

In the present research, our team determined 31 DEGs between BC specimens and nontumor specimens. Then, the outcomes of KEGG analyses unveiled that 31 DEGs were predominantly related to PPAR signal path, AMPK signal path, glycerolipid metabolism, adipocytokine signaling pathway, phenylalanine metabolism, tyrosine metabolic process, and glycine, serine, and threonine metabolic process, highlighting their regulatory function on tumor progression [19–21]. Moreover, based on TCGA datasets, only four DEGs were identified to be survival-related genes, including CRYAB, DEFB132, MAOA, and RBP4. ROC assays further confirmed that they have a strong ability in screening BC specimens from nontumor specimen. Previously, the expressing level and roles of CRYAB have been discussed in multiple cancers [22, 23]. CRYAB suppresses the migratory and invasive abilities of bladder oncocytes via the PI3K/AKT and ERK signal paths [24]. In addition, the prognostic value of CRYAB was also confirmed in several types of tumors, such as colorectal cancer and gastric cancer [23, 25]. In BC, a previous study reported that CRYAB was a prospective biological marker for the identification of BC sufferers at high risk for early recurrence in the cerebrum, regardless of ER and HER2 status [26]. Monoamine oxidase A (MAOA) is a pivotal enzyme related to the metabolic process of monoamine neural transmitters and the regulation of neural transmission, nerve circuits, and cerebrum functions. MAOA has been extensively researched in the background of neural psychiatric illnesses like depression. The expression of MAOA has been discovered to be high in prostate cancer and its overexpression in prostate oncocyte perineural aggression via SEMA3C/PlexinA2/NRP1-cMET signal transmission [27]. However, its function in BC was rarely reported. Retinol-binding protein 4 (RBP4) belongs to the lipocalin family and the main transportation protein of the hydrophobical molecule retinol [28]. A previous study demonstrated a pivotal role of RBP4 in maintaining colon carcinoma self-renewing ability and that such path is a vital link where HFD consumption facilitates colon tumorigenesis [29]. Addition, Wang and his group found that RBP4 is overexpressed in ovarian cancer, and its overexpression promotes cancer the proliferation and metastasis of ovarian cancer cells via regulating RhoA/Rock1 pathway [30]. In BC, RBP4 has been reported to show a diagnostic and prognostic value for BC patients [31]. On the other hand, the potential function of DEFB132 was rarely reported. More experiments were needed to explore its effects on tumor progression.

RETRACTED

To further study whether CRYAB, DEFB132, MAOA, and RBP4 exhibited a dysregulated level in BC, we performed RT-PCR to determine their expression in four BC cells. Interestingly, we only found that the expression of CRYAB and RBP4 was distinctly downregulated in BC cells compared with normal breast cells. Afterwards, our team completed CCK-8 experiments to investigate their roles, discovering that only RBP4 overexpression remarkably repressed the proliferative ability of BC cells. The discoveries of the present research revealed that RBP4 can be an oncogenesis gene in BC development. However, some limitations of this study should be noted. First, every case in the present research was studied retrospectively, and the verification of prospective specimens remains necessary. Second, the specific function of 31 DEGs on several tumor-related pathways has not been investigated. Third, more in vitro and in vivo experiments were needed to further investigate the roles of four critical genes in the proliferative and metastatic abilities of BC cells.

## 5. Conclusion

Overall, we identified four critical genes (CRYAB, DEFB132, MAOA, and RBP4) which may be utilized as novel diagnosis and prognosis biomarkers for BC sufferers. Functionally, RBP4 overexpression suppressed the proliferation of BC cells. Thus, RBP4 may be utilized as a new treatment target for BC.

## Figures and Tables

**Figure 1:** Determination of DEGs in BC. (a, b) Heatmap and volcanic map showed the DEGs between BC and healthy tissues from GSE29431 and GSE42568 datasets. (c) The overlapping DEGs in GSE29431 and GSE42568 datasets.

RETRACTED

**Figure 2:** GO and KEGG analyses of DEGs. (a) The top 10 enriched BP, CC, and MF terms. (b) KEGG pathways.

**Figure 3:** Identification of survival-related DEGs in BC. (a) Low expression of CRYAB, DEFB132, MAOA, and RBP4 indicated a poor prognosis of BC patients from TGCA datasets. (b) The expressing pattern of CRYAB, DEFB132, MAOA, and RBP4 in BC and healthy tissues on the foundation of TGCA datasets.

**Figure 4:** ROC assays of CRYAB, DEFB132, MAOA, and RBP4 in (a) GSE42568 and (b) GSE29431 datasets.

**Figure 5:** RBP4 was lowly expressed in BC and suppressed the proliferation of BC cells. (a, b) The expressing of CRYAB, DEFB132, MAOA, and RBP4 was examined in four BC cells and HBL-100 cells by the use of RT-PCR. (c) CRYAB and RBP4 were distinctly overexpressed in MDA-MB-468 and BT-549 cells after the transfection of pCDNA3.1-CRYAB and pCDNA3.1-RBP4. (d, e) CCK-8 experiments were used to determine the effects of the overexpression of CRYAB and RBP4 on the proliferation of MDA-MB-468 and BT-549 cells. ^∗∗∗^*P* < 0.001, ^∗∗^*P* < 0.01.

## Data Availability

The data used to support the findings of this study are available from the corresponding author upon request.

## Supplementary Materials

Supplementary Materials Table S1: the list of 31 overlapping genes between GSE29431 and GSE42568 datasets.
